# Deep Transfer Learning for Automatic Prediction of Hemorrhagic Stroke on CT Images

**DOI:** 10.1155/2022/3560507

**Published:** 2022-04-16

**Authors:** B. Nageswara Rao, Sudhansu Mohanty, Kamal Sen, U. Rajendra Acharya, Kang Hao Cheong, Sukanta Sabut

**Affiliations:** ^1^School of Electronics Engineering, Kalinga Institute of Industrial Technology, Bhubaneswar, India; ^2^Department of Radio-Diagnosis, Kalinga Institute of Medical Science, Bhubaneswar, India; ^3^School of Engineering, Ngee Ann Polytechnic, 535 Clementi Road, Singapore 599489; ^4^Department of Biomedical Engineering, School of Science and Technology, SUSS University, 463 Clementi Road, Singapore 599491; ^5^Department of Biomedical Informatics and Medical Engineering, Asia University, Taichung, Taiwan; ^6^Science, Mathematics & Technology Cluster, Singapore University of Technology and Design, Singapore

## Abstract

Intracerebral hemorrhage (ICH) is the most common type of hemorrhagic stroke which occurs due to ruptures of weakened blood vessel in brain tissue. It is a serious medical emergency issues that needs immediate treatment. Large numbers of noncontrast-computed tomography (NCCT) brain images are analyzed manually by radiologists to diagnose the hemorrhagic stroke, which is a difficult and time-consuming process. In this study, we propose an automated transfer deep learning method that combines ResNet-50 and dense layer for accurate prediction of intracranial hemorrhage on NCCT brain images. A total of 1164 NCCT brain images were collected from 62 patients with hemorrhagic stroke from Kalinga Institute of Medical Science, Bhubaneswar and used for evaluating the model. The proposed model takes individual CT images as input and classifies them as hemorrhagic or normal. This deep transfer learning approach reached 99.6% accuracy, 99.7% specificity, and 99.4% sensitivity which are better results than that of ResNet-50 only. It is evident that the deep transfer learning model has advantages for automatic diagnosis of hemorrhagic stroke and has the potential to be used as a clinical decision support tool to assist radiologists in stroke diagnosis.

## 1. Introduction

Stroke is the major cause of death worldwide. It occurs when there is interruption in the blood supply to brain parenchyma due to either occlusion (ischemic stroke) or rupture of a blood vessel (hemorrhagic stroke). Intracerebral hemorrhage (ICH), also known as hemorrhagic stroke which occurs when bleeding takes place within the cerebral parenchyma due to rupture of blood vessels. Intracerebral bleed consists of up to 15% of stroke [1] and accounts for 10% of hospital admissions for stroke. It is a challenge to medical fraternity to identify the location of hemorrhage in treating the patient, while ischemic strokes (87%) are more common than hemorrhagic strokes, but within 30 days of onset, the mortality rate is higher in hemorrhagic one [2]. Therefore, rapid diagnosis and posttraumatic treatment are necessary for intracerebral hemorrhage as it is one of the most life-threatening health condition. Imaging techniques like CT and magnetic resonance imaging (MRI) are widely used in detecting stroke. A hyperdense area in NCCT brain suggests hemorrhagic stroke, and also, NCCT brain are cost effective and sensitive for early detection of stroke [3]. Traditionally, classification is done by radiologist by analysis of NCCT brain which is a time-consuming process and error prone. An effective and robust algorithm is needed for automated diagnosis of hemorrhage stroke. Hence, we propose an algorithm based on deep learning which could help the radiologist in decision-making with improved efficiency.

Artificial intelligence (AI) is a recent field of research used for automated detection of brain diseases in CT/MRI images. AI works on large datasets to detect useful patterns that helps in decision-making in disease diagnosis and hence treatment. Machine learning algorithms have been applied successfully for detecting and predicting hemorrhage stroke in NCCT brains [4–7]. Conventional image analysis techniques such as fuzzy *C*-means [8], level set [9, 10], histogram analysis [11], region growing [12], thresholding [13], neural network [14], and random forest [15] have been used to successfully segment the brain hemorrhage. In the thresholding technique, the hemorrhagic lesion is segmented into a region based on threshold of each pixel. Inamdar et al. [7] presented a clustering algorithm using fuzzy *C*-mean and active contour methods to detect the brain hemorrhages. A fuzzy membership degree has been used to control the propagation parameters and to initialize the active contour of the desired object. In a retrospective dataset of 20 CT scans, the method achieved 79% sensitivity, 99% specificity, and an average Jaccard index of 0.78. In a similar work, Bhadauria and Dewal [8] used fuzzy *C*-means clustering to separate the white matter from the skull, and the remaining tissue is separated by the wavelet transform and thresholding. Liao et al. [9] proposed a method for segmenting intracranial hematomas using multiresolution binary level set on brain CT brain images. It works on low-resolution images to improve the efficiency in segmenting the epidural and subdural hematomas. Prakash et al. [10] derived a modified distance regularized level set evolution (MDRLSE) algorithm that improved the speed and detection accuracy in segmenting hemorrhagic lesions. The same method has been used successfully for segmenting brain hemorrhage and its subtypes with an average accuracy of 95% [11]. Subudhi et al. [16] used Delaunay triangulation (DT) with optimization techniques for automatic detecting stroke lesions. The method was effective in accurately segmenting the lesions directly in T2-weighted MRI with less computational complexity. While Ray et al. [17] proposed an intelligent model using the information of pixel distribution and population at different levels to segment hemorrhage in brain CT images. Muschelli et al. [15] used the random forest algorithm to automatically detect hemorrhage regions in CT images; this approach was fast and did not require extensive radiological experience. Indeed, Chung et al. [18] admitted that the standard machine learning approaches are semiautomatic and are not intelligent enough for feature extraction, requiring manual adjustment of parameters to obtain better results and are not suitable for large datasets.

In recent work, CNN-based algorithms have been found to be effective in segmentation classification of medical images [19–21]. Compared to conventional methods, the CNN involves feature extraction through the network itself by observing some pattern in the dataset. Promising results have been obtained by training the CNN models on large dataset to segment brain lesions [22–25]. The first deep CNN architecture, called BrainNetCNN, was presented by Kawahara et al. [26] to predict cognitive and motor developmental outcome in clinical neurodevelopment of infants born networks. They used an automated model based on 3D CNNs refined by a time-implicit multiphase evolution approach to segment abdominal organs. The model is energized by probability map for fine segmentation [27]. In a cascade approach, two 3D patch-wise CNNs are trained to sensitize the lesion voxels, and second model is used to reduce the misclassified voxels. This method was applied for segmentation of white matter (WM) in MRI images of multiple sclerosis (MS) patients [28]. Kamnitsas et al. [29] proposed a computationally efficient method based on deeper CNN model for segmentation of brain lesion by automatic adaptation to imbalance class data. It is a dual pathway, 11 layers deep, and 3D CNN model for simultaneous processing of multiple scale input MRI images. Recently, Wei et al. [30] used a ResNet-based deep learning model to predict celiac disease by analyzing biopsy slides.

Motivated by the goal of providing better diagnosis of brain stroke with limited expertise, we propose a deep learning method focused on reducing error rate. The method is a combined approach consisting of ResNet-50 and dense layer of fully connected layer which incorporates itself a feature extraction method to improve computational efficiency. The residual deep neural network accepts individual CT slices as input, and a fully connected layer classifies the extracted features from the residual network to ICH and normal.

## 2. Materials and Methods

### 2.1. Dataset

We present a retrospective study, where a total of 1164 CT scan images (512 × 512) were collected from 62 patients from both normal (592) and intracranial hemorrhage (572) at the Department Radio-Diagnosis, KIMS under the supervision of radiologists. Noncontrast CT (NCCT) images were acquired by using a 64-slice CT scan machine (GE OPTIMA, 64 slice) having 5 mm slice thickness which were reconstructed to 1 mm slice thickness.

### 2.2. Data Preprocessing

The data preprocessing starts with the extraction of CT slices in DICOM format of size (512,512) and converted to JPG format. A binary image consisting of the skull part in the CT image is extracted with an Otsu's thresholding, and element-wise multiplication operation is performed between the inverted binary image and the CT image to extract the tissue part of the brain with an aim to improve the classification accuracy.

### 2.3. Transfer Learning Model

The proposed framework involves the following steps to classify the head CT images: (1) preprocessing and preparing the input data for the model, (2) automatic discriminative feature extraction using deep residual networks, and (3) classification using fully connected layers as ICH or normal. Deep convolutional neural networks normally extract low-, mid, and high-level features. These extracted features are integrated with the classifiers in a multilayer manner. The performance can be improved by stacking more layers, but this leads to two main problems: vanishing/exploding gradients [31] and performance degradation [32]. However, vanishing/exploding gradients have been addressed in [33, 34]. The performance degradation problem has been addressed in [35], where the authors have introduced a deep residual learning framework called residual network (ResNet).

In ResNet, the stacked layers are trained to fit a residual mapping. Let *H*(**x**) denote the desired mapping and *F*(**x**) denote the residual mapping function where *F*(**x**)≔*H*(**x**) − **x**; **x** is the input to the stacked layer. As shown in Figure 1, the desired mapping *H*(**x**) = *F*(**x**) + **x** can be accomplished by adding shortcut connections into feed forward neural networks.

In ResNet-50 [35], the residual function *F*(**x**) has three convolutional layers, consisting of a layer with 1 × 1 filters, a layer with 3 × 3 filters, and a layer with 1 × 1 filters as illustrated in Figure 1. Each of the above layers is followed by batch normalization (BN) and uses rectified linear unit (ReLU) as activation function. Finally, element-wise addition is performed between the output of the stacked layers (*F*(**x**)) and shortcut connection (**x**). Then, the sum is transited to another ReLU activation function. Shortcut connections of Residual Block1, Block2, Block3, and Block4 in Figure 1 perform identity mapping. The dotted boundary residual blocks in Figure 2 are used to increase the dimensions with a stride of 2 when the shortcut goes across feature maps of two sizes, and a projection shortcut is used to match the dimensions. Transfer learning is a machine learning method where weights (knowledge) of a pretrained model to solve one problem is reutilized to solve another problem [36]. That is, the knowledge gained by the pretrained model is reused for solving target problem.

We use a ResNet-based transfer learning model for the classification of 2D CT images, with a ResNet-50 architecture pretrained on the ImageNet [37] dataset to extract the low-, mid, and high-level features. We then performed classification through the fully connected layers as depicted in Figure 2. After that, the input is convolved with 64 kernels of 7 × 7 size and a stride of 2, followed by max pooling with a stride of 2. The output is then fed to a series of stacked residual blocks followed by a global average pooling (GAP) to reduce the output feature map to 1 × 1 × 2048. These 2048 features are classified by a fully connected layer of 64 neurons, followed by an output layer with a sigmoid activation function. The input head CT image is classified as ICH if the output sigmoid neuron is greater than 0.5; otherwise, it is classified as non-ICH (normal).

### 2.4. Loss Function and Optimizer

The classification of ICH is considered a binary classification problem, where the output label is ICH or normal. So, we use a binary cross-entropy (BCE) loss function for a given input image:

(1) $$\begin{array}{c} L\left(y,\hat{y}\right)=-\left(y\log\left(\hat{y}\right)+\left(1-y\right)\log\left(1-\hat{y}\right)\right), \end{array}$$

where *y* ∈ {0, 1} represents true label for class c and $\hat{y}\in \left[0,1\right]$ represents probability of the predicted observation of class c.

Adaptive moment estimation (Adam) is used as the optimizer for the classification task. Adam unites ideas from root mean square prop (RMSProp) and momentum by computing adaptive learning rates for each parameter.

### 2.5. Evaluation Metrics

The performance and effectiveness of the classification model is demonstrated with the help of accuracy, sensitivity, and specificity measures obtained from the confusion matrix. The performance metrics can be quantified from the confusion matrix as follows:

(2) $$\begin{array}{c} \text{Accuracy}=\frac{\text{TP}+\text{TN}}{\text{TP}+\text{FP}+\text{TN}+\text{FN}}, \end{array}$$

(3) $$\begin{array}{c} \text{Sensitivity}=\frac{\text{TP}}{\text{TP}+\text{FN}}, \end{array}$$

(4) $$\begin{array}{c} \text{Specificity}=\frac{\text{TN}}{\text{TN}+\text{FP}}, \end{array}$$

where TP is true positive, TN is true negative, FP is false positive, and FN is false negative.

## 3. Experimental Results

A ResNet-based transfer learning model was built and used in this paper to classify the CT images as ICH or normal. In this study, two experiments were performed to classify the CT images, first, with only ResNet-50 architecture, and second, with the proposed architecture illustrated in Figure 2, which were pretrained on ImageNet. Before training the two models, the head CT slices were preprocessed, including skull stripping to remove the unwanted regions. Figures 3(a)–3(c) show the positive and negative samples and manually annotated head CT image with ICH lesion, respectively.

After removing the skull part, 512 × 512 × 3 CT images were resized to 224 × 224 × 3 with bicubic interpolation to match with the dimension of the ResNet-50 input layer. Data augmentation is implemented for the generalization of data like horizontal flipping and rotation operations to boost the performance of the proposed model. The two models were trained and tested on 1164 head CT images for 200 epochs with Adam optimizer and BCE as loss function. Out of 1164 CT images, 80% (=931) of the images were used for training the model, and 20% (=233) of the data were utilized for testing the model. The input image of size 224 × 224 × 3 was fed to the 1st layer of convolution where 64 kernels of 7 × 7 were used to filter our input image with a stride of 2, resulting in feature maps of 112 × 112 × 64. The above feature maps were downsampled using 3 × 3 max pooling operations with a stride of 2. Then, the output feature maps obtained were of size 56 × 56 × 64. These feature maps were passed through a series of residual blocks named as Residual Block1, Residual Block2, Residual Block3, and Residual Block4 depicted in Figure 2 to generate the feature maps of 56 × 56 × 64, 28 × 28 × 512, 14 × 14 × 1024, and 7 × 7 × 2048, respectively, followed by global average pooling to give 2048 features. These obtained features were classified using a fully connected layer of 64 neurons and an output layer, with sigmoid activation function, as ICH or normal. The proposed model extracts discriminative features at different layers, and they were used to train the neurons in the dense layers. As can be seen in Figure 4, a sample of feature maps were obtained by propagating the ICH image forward through each block as shown in Figure 2. The performance plots of the two architectures on the head CT scans, like loss vs. number of epochs and accuracy vs. number of epochs, can be seen in Figure 5. The loss and accuracy of the proposed model improved compared to the ResNet-50 model.

The confusion matrices for the two architectures on test data are shown in Figure 6. We achieved 99.6% accuracy, which is about 0.86% more compared to the ResNet-50 model.  Table 1 summarizes the quantitative results in terms of specificity, sensitivity, and area under the curve (AUC), and Figure 7 depicts the receiver-operating characteristics (ROC) on test data. Our results show that the model performed better compared to ResNet-50 alone in terms of measured parameters. Sensitivity refers to the model's ability to correctly detect the patients with ICH, while specificity is the ability of model to correctly find the healthy patients. The sensitivity and specificity of the ResNet-50 model are 0.971 and 0.993, and that of proposed model are 0.994 and 0.997, respectively. The proposed model achieved 1.000 AUC, while ResNet-50 model achieved 0.98 AUC. The time for training the proposed model with 200 epochs is considerably less compared to the other pretrained models, as shown in Table 1. The sensitivity and specificity of the proposed model are improved by adding the fully connected layers to the ResNet-50 model. VGG-16 and GoogleNet are popular deep neural network architectures based on CNNs and trained on ImageNet dataset for ImageNet large-scale visual recognition challenge (ILSVRC). We have also evaluated our dataset with VGG-16 and GoogleNet, achieving comparable results listed in Table 1. Several experiments were conducted with different combinations of hidden layers along with neurons. The results depicted in Figures 5–7 and Table 1 are obtained using the proposed model by taking 64 neurons in the hidden layer of the fully connected layers.

## 4. Discussion

The automated method for detection of intracerebral hemorrhage based on deep learning methods has been summarized in Table 2. Very few algorithms have been reported for automatic detection of ICHs using deep learning approach on CT images. We found a ResNet-based approach used to classify three types of biopsy images with an accuracy of about 90% [30]. Phong et al. [38] adopted the first deep learning approach for detection of intracranial hemorrhage by employing three types of CNN model, i.e., LeNet, GoogLeNet, and Inception-ResNet, and achieved accuracy of 0.99, 0.98, and 0.99, respectively. However, the LeNet model was more time-consuming. Ker et al. [39] proposed a 3D CNN network to classify different hemorrhage types on CT brain images. They applied image thresholding that improved the classification accuracy and measured with better *F*1 scores from 0.91 to 0.95. Lee et al. [40] reported an approach to classify five ICH subtypes from head CT scans collected from 904 cases by using deep learning system and achieved similar performance to expert radiologists with sensitivity of 98% and specificity of 95%. Arbabshirani et al. [41] trained a deep CNN model on nearly 37 thousand hemorrhagic images with AUC of 0.84. They concluded that the deep learning approach can reduce the diagnosis time by 96% in new ICH outpatients. Islam et al. [42] developed an ICHNet for automated ICH segmentation on 3D CT scans where a VGG-16 model was used for training on the data set and classified by 3D conditional random field with Dice accuracy of 87.6%. Chang et al. [43] developed a customized mask R-CNN architecture which uses hybrid 3D/2D version of Feature Pyramid Networks for evaluating hemorrhagic stroke. They quantified the ICH volume with high accuracy measured by Dice score coefficients (0.772-0.931) and Pearson correlations (0.95-0.99). Ker et al. [39] classified CT data into normal and abnormal subtypes using 3D CNN. The *F*1 score of the model for 2-class classification ranged from 0.92 to 0.95. Dhar et al. [44] validated the deep learning algorithm on 224 CT images collected from 124 patients having supratentorial intracerebral hemorrhage. They obtained the accuracy of 98% and suggested for use as a biomarker for rapid quantification of the disease biology in large cohorts. Another study is done by McLouth et al. [45] for validating a deep learning-based tool using 1192 CT images collected from different hospitals for detecting ICH. This tool achieved an accuracy of 95.6% and hence can assist radiologists in emergent detection of ICH lesions in clinical practices. Ye et al. [46] proposed a joint 3D model consisting of CNN and recurrent neural network (RNN) for detecting ICH and its subtypes in noncontrast CT scans of brain in a large dataset consists of 76,621 collected from 2836 subjects from various hospitals. They obtained superior results with an accuracy of 99% in classifying ICH and normal lesions at faster rate; thus, the method has potential to assist radiologists in diagnosis.

Few research works applied U-Net-based fully CNN model with autoencoder for segmenting ICH. Hssayeni et al. [47] used the standard U-Net model on 82 CT scans to segment ICH lesions and achieved a Dice coefficient of 0.31. Danfeng et al. [48] used a ICHNet model to segment and classify ICH, achieving an accuracy of 95%. Patel et al. [49] combined a CNN and bidirectional long-short-term memory (LSTM) model that classifies the for ICH with an accuracy of 95%. Li et al. [50] introduced data symmetry into U-Net-based deep learning framework for detecting and segmenting the hemorrhage strokes. It achieved an accuracy of 98.5% that indicates the effectiveness of the model in clinical decision-making process.

## 5. Conclusions

In this paper, we have presented a ResNet-based transfer learning model for 2D head CT image classification as normal or ICH. The deep transfer learning framework consists of ResNet-50 and a dense layer of fully connected layer. A total of 1164 NCCT brain images were collected from 62 patients with hemorrhagic stroke and used for evaluating the model. The model has been used for accurate classification of hemorrhagic stroke in NCCT brain images, which comprises normal images and ICH lesion of different sizes of ICHs. The images were first preprocessed to remove the skull and resized for the input of the ResNet-50 network to extract the features. The feature set was then classified into normal and ICH using a dense layer of CNN network. Our experimental results indicate that the proposed model outperforms the previous models for the classification by a detectable margin with accuracy of 99.6%. As such, it will be viable to implement the proposed model in a computer-aided diagnosis system to reduce the workload of the radiologists with improved efficiency. As part of our future research, we will emphasize on localizing ICH lesion and classifying its subtypes using different transfer learning approaches to reduce the computational complexity with the potential to further improve the accuracy.

## Figures and Tables

**Figure 1:** Residual learning blocks.

**Figure 2:** Proposed model for prediction of ICH lesion.

**Figure 3:** (a, b) Example of ICH region (positive sample), skull stripping, and manual annotation. (c) Example of negative sample (no ICH region) with skull stripping.

**Figure 4:** Feature maps generated after (a) 7 × 7 conv block, (b) max pool, (c) last Residual Block1, (d) last Residual Block2, (e) last Residual Block3, and (f) last Residual Block4.

**Figure 5:** Performance plots generated on the test set. Plot (a, b) accuracy and loss vs. no. of epochs for ResNet-50 model and (c, d) accuracy and loss vs. no. of epochs for the proposed model.

**Figure 6:** Confusion matrix for ResNet-50 model (a) and proposed model (b).

**Figure 7:** ROC curve and AUC results on the test set for (a) ResNet-50 and (b) the proposed model.

**Table 1:** Comparison of performance measures proposed transfer learning models.

Method	Accuracy	Sensitivity	Specificity	AUC	Training time (sec)
VGG-16	0.931	0.912	0.931	0.965	1849
GoogleNet (InceptionV3)	0.989	0.974	0.986	0.988	1809
ResNet-50	0.982	0.971	0.993	0.984	1835
Proposed model	0.996	0.994	0.997	1.000	1814

**Table 2:** Overview of related work on classification of ICH using CT scans.

Author	Dataset	Method	Performance (%)
Wei et al. [30]	212	ResNet	Accuracy 95.3
Arbabshirani et al. [41]	46583	CNN	Accuracy: 84
Chang et al. [43]	536255	3D/2D mask R-CNN	Sensitivity: 95
Dhar et al. [44]	224	Deep learning	Accuracy: 98
McLouth et al. [45]	1192	Deep learning	Accuracy: 95.6
Danfeng et al. [48]	1176	Fully CNN	Accuracy: 95
Patel et al. [49]	1554	CNN-RNN	Accuracy: 96
Li et al. [50]	159	U-Net	Accuracy: 98.5
Proposed model	1164	ResNet-50 and dense layer	Accuracy: 99.6 Sensitivity: 99.4

## Data Availability

The data used to support the findings of this study are available from the corresponding author upon request.
